# Personality Privacy Protection Method of Social Users Based on Generative Adversarial Networks

**DOI:** 10.1155/2022/2419987

**Published:** 2022-04-13

**Authors:** Yi Sui, Xiujuan Wang, Kangfeng Zheng, Yutong Shi, Siwei Cao

**Affiliations:** ^1^Faculty of Information Technology, Beijing University of Technology, Beijing 100124, China; ^2^School of Cyberspace Security, Beijing University of Posts and Telecommunications, Beijing 100876, China

## Abstract

Obscuring or otherwise minimizing the release of personality information from potential victims of social engineering attacks effectively interferes with an attacker's personality analysis and reduces the success rate of social engineering attacks. We propose a text transformation method named PerTransGAN using generative adversarial networks (GANs) to protect the personality privacy hidden in text data. Making use of reinforcement learning, we use the output of the discriminator as a reward signal to guide the training of the generator. Moreover, the model extracts text features from the discriminator network as additional semantic guidance signals. And the loss function of the generator adds a penalty item to reduce the weight of words that contribute more to personality information in the real text so as to hide the user's personality privacy. In addition, the semantic and personality modules are designed to calculate the semantic similarity and personality distribution distance between the real text and the generated text as a part of the objective function. Experiments show that the self-attention module and semantic module in the generator improved the content retention of the text by 0.11 compared with the baseline model and obtained the highest BLEU score. In addition, with the addition of penalty item and personality module, compared with the classification accuracy of the original data, the accuracy of the generated text in the personality classifier decreased by 20%. PerTransGAN model preserves users' personality privacy as found in user data by transforming the text and preserving semantic similarity while blocking privacy theft by attackers.

## 1. Introduction

Cyberspace threats often focus on a target person to gain access to systems. Social engineering attacks (SEA) using psychological weaknesses of targeted individuals are extremely effective and cause huge losses. Attackers develop a deeper understanding of the target person by discovering psychological attributes of the target with the help of data mining and artificial intelligence, greatly improving the attack success rate. This general approach is shown in Figure 1. However, current defenses against SEA focus nearly exclusively on phishing, even though there are technical means to defend against social engineering attacks. These defenses offer insufficient protection.

Fundamentally, current defense technologies mainly consider only the information characteristics of the attack rather than the characteristics of the targeted person, which makes the defense method too passive. Different targets vary greatly in their vulnerability to SEA, and these differences alter attackers' methods. An important prerequisite for effective SEA protection is determining how attackers find targets' weaknesses.

Human behavioral analysis involves complex psychological factors. Among many psychological factors, personality is a relatively stable and comprehensive psychological feature. Personality has been widely used in security research, and it is an important part of SEA. It is realistic and feasible to make personality the starting point for research into social engineering.

Social media is a key place where individuals share their lives and opinions, with the user's text data open and accessible. This information, when analyzed using machine learning, deep learning algorithm [1, 2], provides effective and accurate personality information from users' own disclosures. Protecting such personality markers effectively inhibits an attacker's ability to perform personality analysis and reduces the success rate of SEA. At present, research into personality privacy protection is nonexistent. Therefore, protecting individual personality data is an appropriate starting point for preventing SEA.

We propose a user personality privacy protection method named PerTransGAN, using generative adversarial networks (GANs) to increase the privacy of user personality data at the source via text transformation and block the theft of personality information. Our contributions are as follows:

1. We design semantic and personality modules in the original GAN framework, the content retention degree of the generated text is improved, the personality information of the original data is transformed, and the classification accuracy of the generated text in the personality classifier is further decreased.
2. We add a penalty term to the loss function of the generator to suppress the weight of words that contribute more to personality information in the real text, to increase the personality difference between source data and synthetic data and reduce user privacy in synthetic text.
3. In addition, compared with the existing model in the field of text generation, including SeqGAN and FGGAN, the generator is added self-attention module to enhance the matching degree between the generated sentence and the real sentence and improve the quality of the generated text.

The rest of this paper is organized as follows. In Section 2, we discuss related work of personality transformation based on text generation. We present our user personality privacy protection model in Section 3. In Section 4, we present and analyze the results of our simulation experiments. Finally, Section 5 presents our conclusions and plans for future work.

## 2. Related Work

The advent of the era of big data has not only promoted the rapid development of science and technology but also exposed user data to all kinds of cyberspace. In order to avoid threats and violations of users' rights and interests and personal privacy, it is very important to study effective privacy protection methods. Wang et al. [3] proposed the framework for cross-silo Federated Learning with Local Differential Privacy (LDP) mechanism, which can provide strong data privacy protection while still retaining user data statistics to preserve its high utility. Radoglou-Grammatikis et al. [4] applied machine learning and reinforcement learning to the modeling of intrusion detection and prevention system, which effectively improved the detection accuracy.

The openness and accessibility of user text data have promoted research into personality information using machine learning and deep networks. It is also a primary source for obtaining user personality data needed for SEA. However, there are no protection methods or related research for personality data.

Using source data, we generate synthetic text that differs from the personality information contained in the source data. This prevents attackers from analyzing the text to determine actual personality information and blunting the attacks. Therefore, text generation and text style transfer (TST) methods are closely related to our work.

Most text generation tasks in the field of natural language processing employ supervised learning for specific applications such as machine translation, speech recognition, and text summary extraction. Unsupervised text generation that estimates the distribution of real text from a text corpus is challenging but more universal. A typical method is to use an encoder-decoder architecture using a recurrent neural network (RNN) [5] to encode the latent representation of sentences and map them into text from the latent space. However, the encoder-decoder architecture usually learns only a limited and structured hidden space, and it is impossible to generate meaningful text from arbitrary latent representations. The probability distribution of latent variables of variational autoencoders [6] also has limitations.

In recent years, GANs have been gradually applied to the field of text generation [7]. GANs introduce an adversarial game between the generator and the discriminator to match the distribution of synthetic and real data and effectively alleviate the problem of exposure bias. However, the discrete nature of the text makes the model nondifferentiable, which hinders the use of GANs in natural language processing tasks.

Solutions to this difficulty are roughly divided into two categories. The first combines a GAN with reinforcement learning (RL), which employs a text generation framework as a sequential decision-making process. Specifically, the gradient of the generator is estimated by a strategic gradient algorithm, such as SeqGAN [8], RankGAN [9], LeakGAN [10], or MaskGAN [11]. The second uses the original GAN framework without RL collaboration. TextGAN [12] and GSGAN [13] use the soft-argmax operator and Gumbel softmax technique [14] to provide continuous approximation on the discrete distribution of the text. Therefore, the model is end-to-end differentiable and provides a low variance gradient for the optimizer, improving the stability and training speed.

Training a GAN to generate text samples involves several challenges. When the discriminator is close to a local optimum, the vanishing gradient leads to an insufficient learning signal from the generator. In addition, mode collapse easily occurs in the training process. TextGAN [15] introduces maximum mean discrepancy (MMD) and reconstruction loss to improve the generator's ability by forcing the empirical distribution of real and synthetic sentences to have matched moments in the latent feature space to alleviate the mode collapse.

In addition to its application in the field of text generation, confrontation training can also be used for text style transfer. Fu et al. [16] proposed a framework to implicitly separate the content and style in text using adversarial learning. After the encoder learns the latent content representation of the input text, two methods are used to generate the text of the target style. One method trains multiple decoders for different styles of output. The second method trains a style of embedding and connects it to the content representation.

However, the preceding adversarial learning TST framework has limitations. Individual style labels may lack content representation, leaving it unable to generate fluent sentences that meet the target style. Therefore, the original method is improved by adding different types of losses. For example, reconstruction loss and cycle-consistency loss have been introduced to improve the content preservation and original style similarity of the TST process [17, 18]. Chen et al. [19] proposed the feature mover GAN (FM-GAN) algorithm to improve the cyclic consistency loss by minimizing the feature-movers distance between the latent representation of the source and the generated sentence.

The preceding research belongs to the strategy of implicit style-content disentanglement. The model needs to learn the content representation and target style embedding of a given text [20]. Recent studies have shown that it is difficult to evaluate the quality of text style-content disentanglement [21]. Therefore, with the help of confrontation learning, reinforcement learning, and probability modeling, newer TST research explores implementations that do not perform style-content disentanglement of the text.

Luo et al. [22] employed two seq2seq models between source and target styles through reinforcement learning without disentangling between style and content. Luo et al. believe that learning the source-target style and target-source style is a dual task. The style classifier reward and reconstruction reward encourage style transmission accuracy and content preservation, and their harmonic averages are used as feedback signals to guide learning. Gong et al. [23] proposed a generator-evaluator architecture using reinforcement learning. The generator uses an attention-based encoder-decoder to transfer styles and a discriminator for adversarial training. It scores the style, content preservation, and fluency of the generated text.

## 3. Materials and Methods

In this paper, we use text transformation to increase personality privacy in user data at the source and prevent privacy theft by attackers. We adopt a GAN architecture and design the semantic and personality modules to protect the personality privacy under the condition of the text similarity. This model consists of four parts: generator *G*, discriminator *D*, the semantic module, and the personality module. The overall network structure is shown in Figure 2.

The process of model training is as follows: firstly, generator *G* takes random token as the starting point of text generation task and uses LSTM to generate each token in the sequence step by step. And with the help of the semantic features extracted by a self-attention mechanism in the real sequence, the generator improves the semantic similarity between the generated sentence and the source sentence.

Then, in the GAN framework, the authenticity of the generated sequence is improved with the help of discriminator D. Therefore, it is necessary to input the sentence from the generator *y*_1_, *y*_2_,…, *y*_*t*_ and real data into the discriminator with the help of the Monte Carlo sampling complement sequence, so as to judge the authenticity of the sequence and output the probability *D*_*ϕ*_ of whether it is real data. At the same time, the advanced features extracted by CNN from the sequence will also be processed by the feature guidance module and transferred to the generator to enhance the text generation process.

In addition, the completed sequence through Monte Carlo sampling will also be input into the personality module and semantic module, respectively, to calculate the personality distance and semantic distance between the real sentence and the generated sentence. Finally, the output probability *D*_*ϕ*_, semantic similarity score *J*_*sem*_, and personality distribution distance *J*_*pers*_ are fed back to the generator, the weighted average of the three is used as a reward signal of reinforcement learning to guide the generator's learning, and the Monte Carlo search is used to pass back to the intermediate state-action step until a complete sequence is generated. The generator adopts the strategy gradient to maximize the feedback reward signal.

## 4. Generator

Generator *G* consists of a text generation module and a semantic guidance module, both of which employ a long-short term memory (LSTM) network structure. The text generation module uses the random token as the initial value and accepts the embedding vector as the LSTM input. According to the specified text length *sequence_ length* *=* *t*, the predicted values at each time step are generated one by one, and the output of the previous time step is used as the input of the next time step. Combined with the semantic guidance module (detailed in the Discriminator), the generation process of the *t*-th time step in the text generation module is shown in (1) and (2):

(1) $$\begin{array}{c} h_{t}=G_{\theta }\left(h_{t-1},x_{t}\right), \end{array}$$

(2) $$\begin{array}{c} q_{t}=W\left(h_{t}w_{t}\right)+c, \end{array}$$

where *θ* denotes the generator parameters, *h*_*t*−1_ is the hidden state of the previous time step, and *x*_*t*_ represents the input vector of the current time step. The hidden state output *h*_*t*_ of the current time step is combined with the guidance vector *w*_*t*_ generated by the feature guidance module. *W* and *c* are the weight matrix and bias coefficient, respectively, in the linear transformation.

In order to ensure that the synthetic sentence matches the real sentence and to improve the semantic similarity, we feed the source text to the token encoded at each LSTM time step after being processed by the self-attention mechanism and use the attention mechanism to integrate the semantic features at each position of the real sentence, as shown in Figure 3.

Due to the lack of location information in the self-attention mechanism, we add the real sequence after word embedding to the positional encoding *PE* with the same dimension and then apply the self-attention mechanism to extract the semantic feature *sem* as shown in (3) and (4):

(3) $$\begin{array}{c} s=x^{r}+PE, \end{array}$$

(4) $$\begin{array}{c} sem=\text{soft}\max\left(\frac{Q\cdot K\_{\text{self}}^{T}}{\sqrt{{\text{d}}_{k}}}\right)\cdot V\_\text{self}. \end{array}$$

In the self-attention mechanism, the query, key, and value vectors should be the text vectors processed by the embedding layer, but the value of the weight matrix for the linear transformation is different and has dimensions d_*k*_. The definition of positional encoding uses sine and cosine functions of different frequencies as proposed by Vaswani et al. [24], and the parameters' description partly reproduces their wording:

(5) $$\begin{array}{c} PE_{\left(pos,2i\right)}=\sin\left(\frac{pos}{10000^{2i/{\text{d}}_{k}}}\right),\\ PE_{\left(pos,2i+1\right)}=\cos\left(\frac{pos}{10000^{2i/{\text{d}}_{k}}}\right), \end{array}$$

where *pos* is the position and *i* is the dimension; that is, each dimension of the positional encoding corresponds to a sinusoid, and the wavelength forms a geometric series from 2*π* to 10000 · 2*π*. After the self-attention layer, the feedforward connection layer and normalization layer deepen the fitting degree of the semantic features by the attention mechanism and normalize values within a reasonable range. In the *t*-th time step, the process of integrating the token encoded by the LSTM into the semantic information at each position in the real sequence is shown in (6) and (7):

(6) $$\begin{array}{c} \alpha_{t}=\text{softmax}\left(\frac{q_{t}\cdot K^{T}}{\sqrt{\text{d}}}\right),\left(K=sem\cdot w^{k}\right), \end{array}$$

(7) $$\begin{array}{c} att_{t}=\sum_{i=1}^{T}\alpha_{ti}V_{i},\left(V=sem\cdot w^{v}\right). \end{array}$$

Similar to the self-attention value, the key and value vectors should be the semantic features *sem* extracted by the self-attention mechanism of the real sequence, and the query vector should be the token encoded by the LSTM in the current time step. The attention weight is calculated according to the information contribution of the semantic features of *t*-th character in the real sequence. After integrating the information, the *t*-th character is resampled by the softmax function.

(8) $$\begin{array}{c} P\left(\cdot |x_{1},\cdots ,x_{t}\right)=z_{t}\left(att_{t}\right)=\text{soft}\max\left(W\cdot att_{t}+c\right),\\ y_{t}∼P\left(\cdot |x_{1},\cdots ,x_{t}\right). \end{array}$$

Through the softmax layer, the probability distribution *z*_*t*_ of the current time step is calculated, and the token *y*_*t*_ is sampled from the probability distribution *P*(·*|x*_1_, ⋯, *x*_*t*_).

## 5. Discriminator

The discriminator *D* uses a convolutional neural network (CNN) structure. First, the input data is vectorized through the word embedding layer. Then, the word vector is fed into the convolution layer, with the text features extracted using convolution kernels of different sizes. Then, the text features are sent to the output layer after being processed by the full connection layer. The output layer uses the softmax function. The discriminator *D* is trained using negative samples generated by the generator *G* and positive samples in the training dataset, which is essentially a binary classification task. For each sample *x*, the discriminator *D* outputs the probability *D*_*ϕ*_(*x*) of sample *x* being real data and feeds it back to the generator *G* as a reward signal in reinforcement learning. The calculation process of the probability value is shown in

(9) $$\begin{array}{c} D_{\phi }\left(x\right)=\text{softmax}\left(\phi_{o}F\left(x\right)\right). \end{array}$$

The optimization objectives of the discriminator *D* are

(10) $$\begin{array}{c} \underset{\phi }{\text{max}}E_{Y∼P_{\text{data}}}\left[\log\;D_{\phi }\left(Y\right)\right]+E_{Y∼G_{\theta }}\left[\log\left(1-D_{\phi }\left(Y\right)\right)\right], \end{array}$$

where *ϕ* denotes the parameter set of the discriminator *D*, *ϕ*_*o*_ denotes the parameters of the output layer, *F* denotes the parameters of the feature extraction network which contain the convolution and pooling layers in the discriminator *D*, and its output *f*_*t*_ is the hidden feature extracted by the CNN that also serves as the input of the semantic guidance module of the generator *G*.

The generator only uses scalar values to optimize the training so that the guidance signal is weak. There is no intermediate syntax structure and semantics to guide the generator to learn fully, so the generator is unable to optimize the network parameters effectively. Therefore, we add a semantic guidance module to the generator network to obtain a richer semantic structure from the discriminator *D* to guide the generation process. In the discriminator *D*, a CNN extracts the context features *f*_*t*_ of the text sequence. The vector is transformed by the LSTM network to obtain the semantic guidance vector to maintain consistency with the feature structure of the text generation module. The process is shown in equation (11).

(11) $$\begin{array}{c} w_{t},h_{t}{}^{C}=C_{\theta_{c}}\left(f_{t},h_{t-1}^{C}\right), \end{array}$$

where *C* represents the semantic guidance module, *f*_*t*_ is the context feature extracted by CNN in the discriminator *D*, *θ*_*C*_ is the parameter set of the semantic guidance module, *h*_*t*_^*C*^ represents the hidden state vector of the current time step in the semantic guidance module, and *w*_*t*_ represents the feature guidance vector converted by the semantic guidance module *C*. In addition, the guidance vector is linearly transformed to ensure the consistency of feature dimensions.

## 6. Semantic Module

In order to hide personality information through text transformation, it is important to preserve the content of the original text to the greatest extent possible in order to establish semantic similarity between the synthetic and real texts. There are many ways to calculate semantic similarity; the cosine similarity, the Jaccard similarity coefficient, and the word mover distance (WMD) are all useable. In addition, deep neural networks can also be used to build the semantic similarity model, as with siamese_LSTM [25], Deep Structured Semantic Model (DSSM) [26], and BERTScore [27].

The selected calculation method must guarantee accuracy but must also reduce computational complexity and avoid performance degradation. We use WMD in the semantic module to measure the semantic difference between synthetic text d^*f*^ and the real text d^*r*^. We use the word shift distance divided by the sequence length as the semantic score. The definition is shown in

(12) $$\begin{array}{c} J_{sem}=-\frac{wmd\left({\text{d}}^{f},{\text{d}}^{r}\right)}{\text{sequence}\_\text{length}}=-\frac{\underset{U\geq 0}{\text{min}}\sum_{i,j=1}^{T}U_{ij}c\left(i,j\right)}{T}, \end{array}$$

where *U*_*ij*_ represents the connection weight between the word *i* in the synthetic text d^*f*^ and the word *j* in the real text d^*r*^ and *c*(*i*, *j*) represents the distance of the word embedding vector between the word *i* and the word *j*. We use the Google pretrained Word2Vec embedding model, which has been trained on a large-scale corpus, to improve the training results and accuracy.

## 7. Personality Module

We use the text transformation method to reduce the available personality information in the user data at the source and calculate the personality difference score between the source and generated texts through the personality module. The personality module learns the personality distribution of the input sequence and uses the Wasserstein distance to measure the distribution distance between two samples. The personality information within the source data is transformed by maximizing the distribution between the real and synthetic texts. The Wasserstein distance is defined as the minimum cost required to transform one probability distribution *P*_1_ into another distribution *P*_2_, as shown in

(13) $$\begin{array}{c} J_{pers}=W\left(P_{1},P_{2}\right)=\underset{\gamma ∼\prod^{}\left(P_{1},P_{2}\right)}{inf}{Ε}_{\left(x,y\right)∼\gamma }\left[\left\|x-y\right\|\right]. \end{array}$$

Compared with the Kullback–Leibler (KL)/Jensen–Shannon (JS) divergence, where the support sets of the two distributions overlap very little, if at all, the Wasserstein distance still reflects the distance between the two distributions. However, the KL/JS divergence is a meaningless value [28]. When the synthetic data are far from the real data, the KL/JS divergence causes the vanishing gradient problem, but the Wasserstein distance continues to provide a smoother result for the parameter updates of the gradient descent.

## 8. Reinforcement Learning

While the goal of the GAN is to generate discrete token sequences, it has some limitations. Most importantly, the discrete output of the generative model makes it difficult to transfer the gradient update from the discriminant model to the generative model. In addition, current deep neural networks only approximate a continuous mapping, but transmission mapping is inherently discontinuous. If the support set of the target probability measure has multiple connected branches, and the continuous mapping is obtained from GAN training, the resulting value domain of the continuous mapping may be concentrated in a connected branch that causes a mode collapse.

In order to solve these defects and implement the transformation of the text data, we “leak” hidden semantic features from the discriminator *D* to the generator *G* to improve the semantic similarity of the generated text. Simultaneously, we add the semantic similarity and personality difference score between the feature vector of the real and generated sentences to the original objective function of GAN to improve the diversity of the generated samples. The sequence generation process is combined with reinforcement learning as a series of action selection, in which the strategy gradient is used to solve the nondifferentiable problem of GAN for text discreteness.

Because the discriminant model can only evaluate a complete sequence, we supplement the incomplete sequence using Monte Carlo sampling, which requires a large number of sampling operations to be carried out in the intervening time to fill the incomplete sequence. The complete sequence *Y*_1:*T*_ is then sent to the discriminator *D* to determine the reward of the current token, and the subsequent generation is carried out according to the feedback guidance. The Monte Carlo search process *MC* for sampling *K* times is shown in

(14) $$\begin{array}{c} \left\{Y_{1:T}^{1},\cdots ,Y_{1:T}^{K}\right\}=MC\left(Y_{1:T}^{1};K\right), \end{array}$$

where *Y*_1:*T*_^*K*^ represents the complete sequence obtained by the *k*-th sampling. In order to ensure the quality and diversity of the generated text and reduce the calculation cost, we set the *K* value to 4.

The action *a* of each step in the sequence generation process selects the next token *y*_*t*_, *a*_*t*_=*y*_*t*_. The state of each step is a prefix sequence composed of generated words, state_*t*_=*y*_1_, ⋯, *y*_*t*−1_. After completing the last time step, the complete sequence is sent to the discriminator *D*, semantic module, and personality module, in that order. Then, the output probability *D*_*ϕ*_, semantic similarity score *J*_*sem*_, and personality distribution distance *J*_*pers*_ are transferred to the generator G. Finally, their weighted average is used as a reward signal to guide the generator's learning. The Monte Carlo search is used to transfer the intermediate state-action step.

The policy of reinforcement learning is expressed as *G*_*θ*_(*a*=*|*state*P*(*a|state*; *θ*), which gives the probability of taking an action *a* in the state state. The action reward value function is defined as *Q*^*θ*^(state, *a*), which represents the overall reward value obtained by taking action *a* in the state state according to the policy. The scores obtained by *K* sampling are averaged into the average expectation *Q*^*θ*^ of the current token, and the granularity of reward guidance is reduced to the level of word. The calculation method is shown in

(15) $$\begin{array}{c} Q^{\theta }\left(\text{state}=Y_{1:t-1},a=y_{t}\right)=\left\{\begin{array}{c} \frac{1}{K}\overset{K}{\underset{k=1}{\sum }}\left(\mu \cdot \;\log\;D_{\phi }\left(Y_{1:T}^{k}\right)+\nu \cdot J_{sem}+\eta \cdot J_{pers}\right),Y_{1:T}^{k}\in MC\left(Y_{1:T}^{1};K\right);t<T\\ \mu \cdot \;\log\;D_{\phi }\left(Y_{1:t-1}\right)+\nu \cdot J_{sem}+\eta \cdot J_{pers};t=T \end{array}\right\}, \end{array}$$

where *μ*, *ν*, and *η* are the weights of the probability score of the discriminator *D*, semantic similarity score *J*_*sem*_, and personality difference score *J*_*pers*_, respectively. The weight value can be adjusted according to the objective function of the generator G. In order to weigh the influence of three signals, we set the weight values as follows: *μ*=0.5, *ν*=0.5, and *η*=1. The total reward expectation *J*(*G*_*θ*_) is defined as

(16) $$\begin{array}{c} J\left(G_{\theta }\right)=E_{Y_{1:T}∼G_{\theta }}\left[Q^{\theta }\left(Y_{1:T-1},y_{T}\right)\right]=\underset{y_{1}}{\sum }G_{\theta }\left(y_{1}|{\text{state}}_{\text{0}}\right)\cdots \underset{y_{T}}{\sum }G_{\theta }\left(y_{T}|Y_{1:T-1}\right)Q^{\theta }\left(Y_{1:T-1},y_{T}\right). \end{array}$$

The goal of the generator *G* is to adopt the strategy gradient to maximize the feedback reward signal, and the loss function of the generator *G* should define the negative value of the reward signal; that is, *L*_*G*_(*θ*)=−*J*(*G*_*θ*_). The gradient descent algorithm of the generator loss is defined as

(17) $$\begin{array}{c} \nabla_{\theta }L_{G}\left(\theta \right)=-\overset{T}{\underset{t=1}{\sum }}\nabla_{\theta }P_{\theta }\left(y_{t}|{\text{state}}_{t}\right)Q^{\theta }\left({\text{state}}_{t},y_{t}\right), \end{array}$$

where ∇ represents the gradient descent process during backpropagation and the parameters *θ* of the generator *G* are adjusted during the process until the loss value converges. *P*_*θ*_(*y*_*t*_*|*state_*t*_) indicates the probability of selecting the next token *y*_*t*_ under the conditions of the state state_*t*_ of the *t*-th step and parameter *θ*.

## 9. Additional Penalty Term

In order to reduce the personality information disclosed in the source data, the key information that plays a decisive role in personality analysis should be reduced or removed from the text. The attention mechanism in deep learning selects the focus position from a large number of pieces of information to produce a more discriminative feature representation. The attention weight coefficient is used to emphasize or select the important information of the target object and to suppress some irrelevant details. As shown in Figure 4, the attention weight distribution of each word in the sentence on a single personality label is inhomogeneous, and the attention weight of the same word on different personality labels is also unequal.

In order to achieve the purpose of personality privacy protection, synthetic data should remove or replace the information related to the users' personality privacy as much as possible. In the personality classification task, the higher the attention weight, the stronger the correlation between the word and personality information, as shown in “nocturnal” in Figure 4. The attention module is designed in the generator to improve the semantic similarity between the generated text and the real text but also to reduce the impact of the key factors of personality privacy in the source text on the synthetic data. Therefore, we set penalties to suppress the corresponding attention weight [29].

We constructed a personality prediction model using a bidirectional long-short term memory (Bi-LSTM) network and attention mechanism to obtain the attention weight matrix in the source data. If the element in the weight matrix is greater than the set threshold *δ*, the text information at the corresponding position shall be punished. We define mask *m* as a binary vector with dimension *T* as

(18) $$\begin{array}{c} m_{i}=\left\{\begin{array}{cc} 1, & \text{if }{Μ}_{i}>\delta ,\\ 0, & \text{otherwise}. \end{array}\right. \end{array}$$

*α* ∈ [0,1] is the attention weight assigned to the sequence feature encoded by the LSTM for each word in the real text in the text generation module of the generator *G*, and ∑_*i*_*α*_*i*_=1. For the loss function *L*_*G*_ of the generator *G*, we add a penalty term Γ to suppress the attention weight of the source text information that plays a key role in personality prediction. The resulting loss function is redefined as *L*_*G*_′=*L*_*G*_+Γ, with

(19) $$\begin{array}{c} \Gamma =-\lambda \text{log}\left(1-\alpha^{T}m\right), \end{array}$$

where *λ* is the penalty coefficient, which is used to adjust the attention value assigned to each sequence feature.

## 10. Results and Discussion

### 10.1. Dataset

We used experimental data from the MyPersonality dataset [30], which includes social data from 250 Facebook users with approximately 10,000 statuses, in which the given personality label is based on the Big Five personality model. It is a complete dataset of social network users, including user text information and external information (such as the time of posting and network size). We used plain-text data from MyPersonality, termed myPersonality_text, and removed the users' external information.

In order to expand the corpus of the model for training and improve the generation ability of the model, in addition to the personality dataset myPersonality_text, we also used the emotional corpus composed of hotel comments collected from the Yelp website [31]. The reviews are classified as either negative or positive. In addition, we took the COCO dataset [32] used for image recognition as real data, which contains the manual text description of each image, to further evaluate the quality of the generated text.

### 10.2. Pretraining

In order to improve the training efficiency and enhance the ability of the model to capture semantic features and personality information in the sequence, we pretrained the generator *G*, discriminator *D*, and personality module.

Generator pretraining: we used maximum likelihood estimation to pretrain the generator *G* and optimize the initial parameters of the generator *G* in order to improve the training speed of the model.

Discriminator pretraining: the discriminator *D* used the cross-entropy loss function for pretraining in order to improve the ability to capture semantic features in the sequence and to enhance the guidance and information within the guidance signal.

Personality model pretraining: the personality module was constructed using Bi-LSTM and an attention mechanism. The samples in the myPersonality_text dataset were used as input so that the model would learn the personality distribution in the social text and train the personality model to predict the personality label.

### 10.3. Evaluation

In this paper, the effectiveness of personality privacy protection methods is verified mainly through the following three aspects.

#### 10.3.1. Text Quality

The BLEU score [33], an evaluation metric for the quality evaluation of the generated text, compares and counts the number of commonly occurring n-ary words to measure the similarity degree between the generated texts and the human-created texts.

BLEU-1 tests whether each word in the real sentence appears word by word in the generated text, while BLEU-2 and above indicators reflect the fluency of the synthetic text. Its value range is between 0.0 and 1.0. The higher the matching degree between two sentences, the higher the BLEU equal score. If two sentences perfectly match, the BLEU score is 1.0.

#### 10.3.2. Content Preservation

In the process of personality transformation, a key requirement is the retention of the content in the source data and the maintenance of the semantic similarity between real and synthetic data. We used the metric proposed by Fu et al. [16]. The strength content preservation is defined as the cosine distance between the source sentence embedding *v*^*r*^ and the synthetic sentence embedding *v*^*f*^:

(20) $$\begin{array}{c} \text{score}=\frac{{\left(v^{r}\right)}^{T}\cdot v^{f}}{\left\|v^{r}\right\|\cdot \left\|v^{f}\right\|}. \end{array}$$

Here, sentence embedding consists of the max, min, and mean pooling of the word embedding, *v*=[*v*_min_, *v*_mean_, *v*_max_]. The embedded model is Word2Vec, which is pretrained by Google. After training it with English Wikipedia, it was adjusted according to the corpus used in the experiment.

#### 10.3.3. Personality Transformation

We established a text generation model using a GAN to reduce personality information disclosed in source data and block SEA. Whether users' personality privacy can be analyzed from social text data was evaluated by the accuracy of the personality classifier, and the reduction of personality disclosure was measured by the change in the personality classification results. The classifier proposed by Wang et al. [1] was constructed using hierarchical attention, CNN, Bi-LSTM, which was trained on the training dataset for personality prediction. If the transformed social text no longer conformed to the original personality label, the accuracy of the trained classifier model would decline.

### 10.4. Content Preservation and Text Generation

In order to verify the performance of the proposed model in text generation, we conducted a comparative experiment on the COCO dataset. The comparison experiment took the BLEU score as the quality evaluation index of the text and compared it with the experimental results of SeqGAN, RankGAN, RelGAN, and FGGAN. The experimental results are shown in Table 1. The experimental data shows that the performance of the PerTransGAN model is better than that of the comparison model, and the quality of the generated text has been improved to a certain extent.

In order to explore the text quality of the PerTransGAN model on different datasets, we calculated the BLEU score of text generated on the MyPersonality dataset. The experimental data are shown in Table 2. It can be seen from Table 2 that the BLEU-3 and BLEU-4 scores on the MyPersonality dataset are higher than those of the COCO dataset, and the performance of the PerTransGAN model in the text generation task is relatively stable.

Our model used the SeqGAN model proposed by Yu et al. as the baseline and added the feature guidance module (Add_FG) designed by Yang et al. In order to enhance the correlation between the synthetic text and the source data, we used the self-attention mechanism (Add_Attention) to integrate the key semantic information in the source data. The experimental data on the MyPersonality dataset in Figure 5 shows that the addition of the feature guidance module and attention mechanism improved the content preservation of the synthetic text. Compared to the baseline model, the preservation strength of the original semantic content was improved by about 0.2.

In addition, a key part of our text generation task was to reduce personality disclosure in text data while ensuring semantic similarity. Therefore, the personality and semantic modules were designed in our text generation model PerTransGAN to enhance the goal diversity of GAN. Similarly, the degree of content preservation was also improved to some extent, from 0.834 to 0.859.

Some typical examples of the sentences generated by our model on the MyPersonality dataset and Yelp restaurant reviews are shown in Table 3. Table 3 shows that, in order to achieve the goal of reducing personality disclosure, the changes in the text information consisted of sentence structure changes, emotion transformations, synonym replacements, and writing style transfer. For example, the phrase text “highly recommended” was added with a subject-predicate structure to synthesize a complete sentence combined with the first half of the source sentence.

In addition, social network users tend to use informal symbols, which may include customized terms of emphasis, overlapping punctuation, and symbolic expressions such as “soooooooo,” “zzz,” “!!!,” and “).” In order to study the effect of these informal symbols on the personality of social users, we reserved these special words when preprocessing the dataset.

A sentence may contain nouns, adjectives, verbs, auxiliary verbs, and adverbs. We believe that, due to the different part of speech and meaning of each word in the sentence, diverse words carry different amounts of personality information, and the contribution of the same word in a sentence to each personality label is also different. Therefore, the attention weight distribution of words in each position on the personality labels is uneven.

Figure 6 shows the attention weights of the keywords in the source sentence and the composite sentence to the five personality labels. Among them, customized special symbols and emotional adjectives have a high weight, which plays a critical role in personality classification. The attention weight of nonreal verbs such as prepositions and be verbs is low, and the numerical difference is small. In the experiment, we found that the text generation results included the addition replace or removal of custom symbols and emotional words, which leads us to believe that there is a relationship between users' writing style and personality information.

### 10.5. Personality Transformation

We divided the myPersonality_text dataset into training and test sets and used the training set to train both the text generation model PerTransGAN and the personality classification model. Then, the test set was fed into PerTransGAN to generate target text, and the personality labels of source and synthetic texts were identified by the trained personality classifier.

In order to verify the effectiveness of the proposed framework PerTransGAN in personality privacy protection, we used the personality classification model HMAttn-ECBiL [1] proposed by Wang et al. to detect the personality information in the source text and the generated text and observed whether the classification accuracy of the model decreases significantly. The first row of data in Table 4 shows the personality classification results of the source text from the test set.

In addition, in order to verify the effectiveness of the penalty term in the objective function in reducing personality disclosure, we set different penalty coefficients for the text generation tasks and removed the personality module of PerTransGAN.

The data in Table 4 shows that the classification accuracy of the text generated by the proposed PerTransGAN model was lower than that of the real text. The results show that the prediction results of the synthetic text no longer accorded with the original personality label, indicating a change in the personality data and a reduction in personality disclosure. The accuracy of personality classification changes slightly when the penalty item is not added (*λ*=0). When the penalty term was added to the objective function, the accuracy of personality classification continued to decline as the penalty coefficient increased. When the value of the penalty coefficient *λ* equaled 1, the decline range of classification accuracy of each personality is the highest and the maximum decreases by 13%.

It can be seen from the data change trend in Table 4 that, with the increase of punishment coefficient, the personality information in the text data has further changed, and the reduction of classification accuracy has increased. However, the semantic content in the original text was also affected, and the degree of content preservation decreased. In the generated text, we find that some sentences changed the original emotional attitude or lost the topic words. Therefore, the punishment coefficient should not be set too large, and it is necessary to compromise between the degree of content preservation and personality transformation.

In order to explore the influence of the personality module on the experimental results, the penalty coefficient of the model is fixed to 0.5. The experimental results are shown in Figure 7, which compared the result change of the PerTransGAN model with or without the personality module. Among them, the average classification accuracy of the HMAttn-ECBiL model to the original data was 72.01%.

Firstly, we conducted a personality classification experiment on the text generated by the model without the personality module. The average classification accuracy was 65.84%. As can be seen from Figure 7, the difference in the classification accuracy compared to the results of the original data was small, which was reduced by about 6%.

The average accuracy of the text generated by the PerTransGAN model with personality module in personality classifier was 55.28%. Moreover, the classification accuracy of the five kinds of personality decreased to varying degrees, and the classification accuracy remained around 55%, of which the accuracy of OPN personality decreased by about 20%. Therefore, on the premise of ensuring semantic similarity, the personality information carried in the text generated by the PerTransGAN model is inconsistent with the real label in the source data, which increases the personality difference so that the attacker cannot obtain the real personality characteristics and achieve the purpose of privacy protection.

## 11. Conclusions

We propose a GAN-based personality privacy protection method called PerTransGAN for social network users that combines with reinforcement learning to transform personality information in source data for the sake of reducing personality disclosure. We modified the baseline model and designed the semantic and personality modules to strengthen the constraints of semantic and personality information within synthetic texts. In addition, we added a penalty term to the objective function to limit the impact of the key information of the source data on the synthetic text in the personality prediction task.

By observing the results of text generation, we found that text modifications largely include sentence structural changes, emotion transformations, synonym replacements, and writing style transfer. There is also a correlation between users' preferred vocabulary, writing style, and personality. Based on the content preservation evaluation metric proposed in previous work and the resulting changes in the personality classifier, we verified the effectiveness of the model. The experimental data shows that, with the addition of the self-attention module and semantic module in the generator, the content preservation degree of the generated text is improved by 0.11 compared with the existing model. In addition, with the addition of the penalty term and personality module, the accuracy of the generated text in the personality classifier is decreased again, which is 20% lower than the original data in the optimal case. The proposed PerTransGAN generates synthetic text that successfully obscures personality information found in the source data, which interferes with the accuracy of personality analysis and thwarts possible attackers.

In future work, we plan to explore the correlation between text style and personality information on the basis of an analysis of our experimental results, starting with the user's writing style as it relates to protecting user personality information.

## Figures and Tables

**Figure 1:** Social engineering attack process using personality information.

**Figure 2:** Overall network structure diagram.

**Figure 3:** The attention mechanism used to fuse the information in the source text sequence.

**Figure 4:** Attention weights of different words in sentences on five personality labels. The change of color from dark to light indicates that the attention weight increases gradually.

**Figure 5:** The degree of content preservation with different model architectures.

**Figure 6:** Attention weights of keywords in source sentences and generated sentences on five personality labels. The change of color from dark to light indicates that the attention weight increases gradually. (a) Source sentence. (b) Synthetic sentence.

**Figure 7:** Model accuracy of personality classification in source data and generated data.

**Table 1:** Comparison of BLEU scores of different models on the COCO dataset.

	SeqGAN	RankGAN	RelGAN	FGGAN	PerTransGAN
BLEU-2	0.734	0.748	0.765	0.773	0.783
BLEU-3	0.519	0.532	0.548	0.559	0.590
BLEU-4	0.371	0.394	0.406	0.417	0.433
BLEU-5	0.237	0.271	0.323	0.359	0.377

**Table 2:** BLEU scores of PerTransGAN model on the MyPersonality dataset.

	BLEU-2	BLEU-3	BLEU-4	BLEU-5
PerTransGAN	0.759	0.609	0.447	0.330

**Table 3:** Example text generation results.

Dataset	Source sentence	Synthetic sentence
MyPersonality	“What's on your mind summer programmmms?” ahhhhhhhhhhhhhhhhhhhhh go go go go go	What summer arrangement that *u* want, perfect programmmms come on
	is bored being back home already	Being back home is excitement time
	Kindly thanks everyone who wished him a happy birthday!	Sooooooo grateful for those who sent him birthday wishes

Yelp restaurant reviews	Our server was one of the friendliest coolest girls that we have ever met	The coolest girl we've ever seen serves us with a smile
	The spelt bun was better than any other spelt bun/bread that I've ever had before	This spelt bread was the best bread I've ever eaten
	Perfect spot for breakfast, lunch or take-out. Highly recommended	This ideal place is highly recommended to choose brunch or take-out

**Table 4:** Comparison of content preservation and classification accuracy of text generation results with different penalty coefficients.

Penalty coefficient *λ*	Content preservation	EXT (%)	NEU (%)	AGR (%)	CON (%)	OPN (%)
—	—	73.94	62.14	70.74	68.65	84.57
0	0.859	71.88	65.38	66.40	63.55	82.38
0.3	0.847	68.57	61.11	65.90	60.54	79.69
0.5	0.824	67.43	60.93	62.54	63.20	75.08
1	0.786	62.65	53.90	57.85	56.03	71.18

## Data Availability

Previously reported MyPersonality data were used to support this study and are available at https://www.psychometrics.cam.ac.uk/productsservices/mypersonality. Previously reported Yelp restaurant reviews data were used to support this study and are available at https://www.yelp.com/dataset. In addition, previously reported COCO dataset was used to support this study and is available at https://cocodataset.org/#download. The prior studies are cited at relevant places within the text as references [30–32].

## References

[1] Wang X., Sui Y., Zheng K., Shi Y., Cao S. (2021). Personality classification of social users based on feature fusion. *Sensors*.

[2] Wu L., Quan C., Li C., Wang Q., Zheng B., Luo X. (2019). A context-aware user-item representation learning for item recommendation. *ACM Transactions on Information Systems*.

[3] Wang C., Wu X., Liu G., Deng T., Peng K., Wan S. (2021). Safeguarding cross-silo federated learning with local differential privacy. *Digital Communications and Networks*.

[4] Radoglou-Grammatikis P., Rompolos K., Sarigiannidis P. (2021). Modeling, detecting, and mitigating threats against industrial healthcare systems: a combined software defined networking and reinforcement learning approach. *IEEE Transactions on Industrial Informatics*.

[5] Cho K., Van M. B., Gulcehre C. Learning phrase representations using Rnn encoder-decoder for statistical machine translation.

[6] Bowman S. R., Vilnis L., Vinyals O., Dai A. Generating sentences from a continuous space.

[7] Goodfellow I. J., Pouget-Abadie J., Mirza M. (2014). *Generative Adversarial Nets*.

[8] Yu L., Zhang W., Wang J., Yu Y. (2017). SeqGAN: sequence generative adversarial nets with policy gradient. *Proc. AAAI*.

[9] Lin K., Li D., He X., Zhang Z., Sun M. T. (2017). Adversarial ranking for language generation. *Proc. NIPS*.

[10] Guo J., Lu S., Cai H., Zhang W., Yu Y., Wang J. (2018). Long text generation via adversarial training with leaked information. *Proc. AAAI*.

[11] Fedus W., Goodfellow I., Dai A. M. (2018). MaskGAN: better text generation via filling in the _. *Proc*.

[12] Zhang Y., Gan Z., Fan K. (2017). Adversarial feature matching for text generation. *Proc. ICML*.

[13] Kusner M. J., Hernández-Lobato J. M. (2016). GANS for Sequences of Discrete Elements with the Gumbel-Softmax Distribution. https://arxiv.org/abs/1611.04051.

[14] Maddison C. J., Mnih A., Teh Y. W. (2017). The concrete distribution: a continuous relaxation of discrete random variables. *Proc*.

[15] Salimans T., Goodfellow I., Zaremba W., Cheung V., Radford A., Chen X. (2016). Improved techniques for training GANs. *Proc. NIPS*.

[16] Fu Z., Tan X., Peng N., Zhao D., Yan R. Style transfer in text: exploration and evaluation.

[17] John V., Mou L., Bahuleyan H., Vechtomova O. Disentangled representation learning for non-parallel text style transfer.

[18] Yin D., Huang S., Dai X., Chen J Utilizing-parallel text for style transfer by making partial comparisons.

[19] Chen L., Dai S., Tao C. (2018). Adversarial text generation via feature-mover’s distance. https://arxiv.org/abs/1809.06297.

[20] Hu Z., Lee R. K., Aggarwal C. C. (2020). Text Style Transfer: A Review and Experiment Evaluation. https://arxiv.org/abs/2010.12742.

[21] Lample G., Subramanian S., Smith E. M., Denoyer L., Ranzato M., Boureau Y. Multiple-Attribute Text Rewriting,” in 7th International Conference on Learning Representations.

[22] Luo F., Li P., Zhou J. A dual reinforcement learning framework for unsupervised text style transfer.

[23] Gong H., Bhat S., Wu L., Xiong J., Hwu W. (2019). Reinforcement learning based text style transfer without parallel training corpus. *Proceedings of NAACL-HLT*.

[24] Vaswani A, Shazeer N, Parmar N Attention Is All You need.

[25] Mueller J., Thyagarajan A. (2016). Siamese recurrent architectures for learning sentence similarity,” proceedings of the thirtieth AAAI conference on artificial intelligence. *Proc. AAAI*.

[26] Huang P., He X., Gao J., Den L., Heck L. Learning deep structured semantic models for web search using clickthrough data.

[27] Zhang T., Kishore V., Wu F., Weinberger K. Q., Artz Y. (2019). Bertscore: Evaluating Text Generation with Bert. https://arxiv.org/abs/1904.09675.

[28] Arjovsky M., Bottou L. (2017). Towards principled methods for training generative adversarial networks. *Proc. ICLR*.

[29] Pruthi D., Gupta M., Dhingra B., Neubig G., Lipton Z. C. (2020). Learning to deceive with attention-based explanations. *Proc. ACL*.

[30] Kosinski M., Matz S. C., Gosling S. D., Popov V., Stillwell D. (2015). Facebook as a research tool for the social sciences: opportunities, challenges, ethical considerations, and practical guidelines. *American Psychologist*.

[31] Shen T., Lei T., Barzilay R., Jaakkola T. (2017). Style Transfer from Non-parallel Text by cross-alignment. https://arxiv.org/abs/1705.09655.

[32] Chen X., Fang H., Lin T.-Y. (2015). Microsoft COCO Captions: Data Collection and Evaluation Server. http://arxiv.org/abs/1504.00325.

[33] Papineni K., Roukos S., Ward T., Zhu W.-J. ‘BLEU: a method for automatic evaluation of machine translation.

